# Psychological Distress Among Women Healthcare Workers: A Health System's Experience Developing Emotional Support Services During the COVID-19 Pandemic

**DOI:** 10.3389/fgwh.2021.614723

**Published:** 2021-02-09

**Authors:** Jesse Sanford, Alpna Agrawal, Karen Miotto

**Affiliations:** ^1^Semel Institute for Neuroscience and Human Behavior, University of California, Los Angeles, Los Angeles, CA, United States; ^2^Department of Psychiatry and Biobehavioral Sciences, Semel Institute for Neuroscience and Human Behavior, University of California, Los Angeles, Los Angeles, CA, United States; ^3^VA Greater Los Angeles Healthcare System, Los Angeles, CA, United States

**Keywords:** women, healthcare worker, mental health, emotional support, wellness, COVID-19

## Abstract

Ensuring the mental health and well-being of the healthcare workforce globally, especially women healthcare workers (HCWs), is an ongoing challenge that has been accentuated by the novel coronavirus (COVID-19) pandemic. Already at high risk of experiencing symptoms of stress, burnout, and depression, women HCWs are now also facing the psychosocial impacts of the COVID-19 pandemic. Although different types of mental health interventions have been introduced to support HCW well-being, the current needs of women HCWs have not been emphasized and replicable processes for developing and implementing specific emotional support services for women HCWs have not yet been well-described in the literature. Therefore, in this perspective, we discuss the approach our institution (University of California, Los Angeles) took for developing emotional support services for women HCWs that incorporate aspects of disaster behavioral health models and address various barriers to support and treatment. In addition, we describe and illustrate the process that we utilized to develop individual-level and institutional-level emotional support services. Finally, based on our institution's experience, we share recommendations for developing emotional support services for women HCWs during the COVID-19 pandemic and other future crises.

The most precious thing I gained from the support I received was to understand the importance of scheduling time for my own self-care and self-compassion. I never realized that I spent most of my life caring for others and very little time on my own needs. The COVID-19 pandemic has brought us to an unpredictable time in history, but I am excited to report my self-care, self-compassion, and elevated level of self-awareness will be a few of my bright spots during this unsettling time.

- Woman healthcare worker who received emotional support services from our institution

## Introduction

Women healthcare workers (HCWs) experience a unique set of work and individual life stressors, often resulting in significant gender-related differences in mental health symptoms and outcomes. Factors that affect women HCWs' well-being include (a) role strain (b) difficulties establishing and maintaining work-life balance, (c) consequences associated with pregnancy and motherhood, (d) gender bias and discrimination, (e) imposter syndrome, and (f) a lack of sufficient support systems (1–4).

These stressors often leave little time or opportunities for self-care or self-compassion, leading to lower levels of self-valuation among women HCWs (5). Moreover, with regards to the effects of these stressors on mental health conditions, in addition to high levels of stress (1), women HCWs experience significantly higher rates of burnout (4, 6, 7) and depression or depressive symptoms than their male colleagues (3, 8).

High rates of mental health problems among women HCWs are particularly worrisome, since HCWs are reluctant to seek regular healthcare for themselves and are often unwilling to engage with mental health treatment. For example, 35% of physicians (9) and nearly 20% of physician assistants (10) do not have an established, regular source of care for receiving preventive healthcare services. Moreover, physicians' use of mental health services is low (11), especially among females, as evidenced by the fact that nearly 50% of women physicians surveyed who believed they met criteria for a mental illness reported not seeking mental health treatment (12). Previous research has suggested that women HCWs frequently cite a lack of time, concerns related to confidentiality and stigma, and fear of professional consequences, including effects on licensure status, as barriers to engaging with mental health services (12, 13). Organizational barriers to accessing supportive services also include decentralized services and employee assistance or mental health treatment programs only offering appointments during normal business hours, impacting women HCWs who are working or assisting with childcare or educational responsibilities.

Recent global large-scale studies, systematic reviews, and meta-analyses examining the mental health outcomes of HCWs during the COVID-19 and prior pandemics have confirmed the aforementioned trends related to gender differences in HCW well-being. For instance, psychological distress during pandemics has been found to be associated with gender (14, 15) and compared to male coworkers, women HCWs reported experiencing higher rates of depression, anxiety, insomnia, and distress (16–23). Finally, considering the fact that barriers to accessing mental health services have likely intensified because of the pandemic, the current state of HCWs'-especially women HCWs'-mental health and well-being, is cause for concern and must be addressed.

Although various interventions to support the mental health of HCWs during the COVID-19 pandemic have been described in the literature (24) and calls to include a gender perspective when developing interventions have been made (25), there remains limited information on the specific needs of women HCWs during this challenging time and specific processes institutions can use to develop and implement emotional support services. Therefore, in this perspective, we (1) briefly review useful disaster behavioral health models that informed the development of emotional support services at our institution (University of California, Los Angeles); (2) present an online interactive screening program that assessed the impact of the COVID-19 pandemic on HCWs and served as a qualitative needs assessment; (3) provide qualitative needs assessment data from women HCWs that we referred to in the development of additional services at both the individual and institutional levels for this population; and (4) outline recommendations for developing emotional support services for women HCWs based on our institution's experience.

## Models of Disaster and Crisis Psychological and Behavioral Health Interventions

When our institution's COVID-19 wellness and mental health workgroup first convened to address HCW well-being during the COVID-19 pandemic, members reviewed disaster behavioral health models. These models subsequently informed the development of our COVID-19 emotional support and mental health response plan for all HCWs (26). Various models have been proposed for supporting individuals during crises or after disasters and while many models share certain aspects, our workgroup identified three models to utilize. One model recommended by the National Academy of Medicine describes a tiered public health approach, consisting of universal resources and information, targeted logistical and psychological interventions, and intensive mental health services. This model allows for triage to an appropriate level of care with tier-specific interventions, services, and resources (27). The second model was Psychological First Aid (PFA), developed by the National Child Traumatic Stress Network and the National Center for PTSD. Key, relevant tenants of PFA include information gathering to identify needs, offering assistance that addresses immediate needs and concerns, and connecting and linking individuals with social supports and other services (28). The third model was a specific set of COVID-19-related institutional recommendations, which also included a list of thematic requests that HCWs may direct toward their respective organizations. We reviewed the themes from the third model and aimed to ensure that our emotional support and mental health response plan for HCWs addressed many of these requests, especially HCWs' appeals to their organizations to feel heard, supported, and cared for during the COVID-19 pandemic (29). In sum, the three models emphasized the importance of conducting a needs assessment, providing emotional support services, and a healthcare system's response to addressing the specific needs of HCWs during crises.

## Development of Emotional Support Services for Women HCWs During the COVID-19 Pandemic

As part of our institution's overall COVID-19 emotional support and mental health response plan (26), we developed a variety of emotional support services for all clinical and non-clinical HCWs. After reviewing the relevant disaster behavioral health models, we conceptualized the flow of services to begin with HCWs accessing an online interactive screening program and providing qualitative data regarding their current psychosocial and mental health needs via a needs assessment. At our institution, as is typically found in mental health intervention research, the majority of participants were women. Therefore, we determined that, based on the feedback we received from women HCWs, we would develop tailored additional services for this population at both the individual and institutional levels. A pictorial description of the development and introduction of these services is outlined below in Figure 1.

**Figure 1:** Our institution's process of developing and introducing emotional support services for HCWs during the COVID-19 pandemic.

### Interactive Screening Program and Embedded Qualitative Needs Assessment

The online interactive screening program was developed in coordination with the American Foundation for Suicide Prevention and designed to both assess COVID-19-related anxiety, depression, and stress, as well as provide all HCWs with an opportunity to express their fears and concerns. The screening program totaled 16 questions, including the 12-item Coronavirus Impact Scale (30) and the 4-item Patient Health Questionnaire (PHQ-4) (31). The Coronavirus Impact Scale measures the extent to which the COVID-19 pandemic has changed one's life across multiple domains, including the following: routines, family income/employment, food access, medical health care access, mental health treatment access, access to social supports, COVID-19-related stress, familial stress/discord, and diagnosis of coronavirus among self, immediate family members, and extended family members and/or close friends (30). The PHQ-4 screens for anxiety and depressive symptoms (31). The qualitative needs assessment was embedded within the interactive screening program and asked program users to indicate (1) how they felt the current situation has impacted their lives, (2) what they were finding most challenging, and/or (3) what support they thought would be most helpful at the time. Since the majority of participants were women, our programmatic response to the needs assessment focused on addressing women HCWs' stressors and devising services specific to this population. Thematic analysis of ~100 women HCWs' responses to the qualitative needs assessment resulted in the discovery of 10 main themes of concerns. The most commonly cited theme was related to workplace dynamics/duties, followed by concerns regarding family/friends, health (physical and emotional), anxiety, work-life balance, stress, finances, education (predominantly of their children), depression, and burnout.

### Individual-Level Support Services

Confidential services available to all women HCWs were delivered by mental health professionals via phone (text, call) or web (email, screening program platform). Specific examples of services provided include hiring trained counselors to (1) engage in sustained, anonymous dialogue with users over the online screening program platform; (2) provide resources for logistical support (e.g., institutional, community, and governmental resources for securing childcare, food delivery, and vouchers for lodging to self-isolate from family members) via phone or web; and (3) via phone or web, refer participants to formal mental health services and assist them as they established care. We also launched an institution-wide emotional support request phone line staffed by mental health professionals (e.g., psychologists and psychiatrists). In addition to those that requested a check-in call after dialoguing with a counselor over the screening program platform, many women HCWs first engaged with our services by texting or calling the line to request an emotional support check-in call.

### Institutional-Level Support Services

Four institutional initiatives related to high-risk units or departments, leadership development, community pods, and parenting forums were designed. Recognizing that any obstacle to engaging with needed support becomes magnified during disasters or crises, we matched high-risk clinical and non-clinical units, departments, or workgroups with mental health clinicians to serve as an embedded designated resource for emotional support and mental health concerns. Depending on their familiarity with their assigned workgroups, these clinicians joined regular, recurring staff huddles or held additional ones to introduce themselves, listen to staff concerns, and normalize the fear and stress associated with adjusting to the implications of new realities. These clinicians also escalated reported concerns to the workgroup leadership team, which resulted in further tailored institutional support. For example, after the embedded clinician for the Emergency Department learned that HCWs were experiencing symptoms of insomnia and sleep disturbances, the workgroup coordinated an educational and supportive session on sleep and insomnia among HCWs during the time of COVID-19. After learning that certain supervisors were finding it difficult to inspire, motivate, and manage their non-clinical HCW teams in the face of prolonged uncertainty and consistently changing protocols, we developed a series of department-specific leadership development courses. These sessions educated supervisors on the tenants of stress first aid and PFA, and provided them with opportunities for peer support and self-reflection in group sessions so that leadership personnel could then model what they experienced in these sessions with their own staff and teams. An additional noteworthy outcome of campus-wide feedback is the formation of community bubbles or pods that enable HCWs' families to connect with other families at our institution for shared childcare, educational opportunities, or socio-emotional experiences either virtually or safely in-person. Finally, parenting forums for all HCWs currently under development will provide content related to child development, child disaster behavioral health, and parenting strategies during disasters and crises. The forums will also offer parents a space to raise questions or concerns. These forums may prove to be especially helpful as many women HCWs' children return to school, albeit via new formats and with an uncharted set of circumstances.

## Discussion

Research shows women HCWs report high levels of psychological distress and more recent studies have shown this trend to remain constant or become exaggerated as a result of the COVID-19 pandemic (32). We found these findings from the literature to be reflected in the demand for emotional support services provided by our organization during the COVID-19 pandemic. As described here, this demand prompted us to focus on addressing the specific needs of women HCWs in our organization.

The significance of incorporating crisis behavioral health models in our work was made explicit by members of our workgroup leadership team, some of whom are experts in the field of disaster psychology themselves and oversee operations at a national center for trauma. Although the emphases of these disaster behavioral health frameworks slightly differ, they are complementary and we utilized aspects of each one in planning our emotional support services. For instance, we utilized the three-tiered approach for determining the levels of care we would provide and the associated level-specific interventions. We used PFA to establish the progression of our interventions, beginning with conducting a needs assessment, followed by offering practical assistance for addressing immediate needs, connection with social supports, and linkage with other services. Finally, throughout our work, we kept in mind the thematically classified requests of HCWs to their organizations during the COVID-19 pandemic to hear, support, and care for them.

The goals of the online interactive screening program were 2-fold: to provide individual-level emotional support and assess the needs of HCWs for future construction of additional individual-level and other institutional-level support services. Moreover, we sought to provide a service that addressed frequently identified barriers to accessing support and treatment among HCWs, including a perceived lack of time and concerns related to confidentiality. Since shorter questionnaires yield higher response rates among HCWs (33), we limited the length of the screening program by asking a total of 16 questions (excluding demographic questions) and utilized the PHQ-4, an abbreviated screening assessment for anxiety and depression. We also conceptualized the screening program to function in a dual capacity, since anecdotal evidence suggests that survey fatigue is already high among HCWs and workgroup members advocated for a time-efficient and streamlined process for HCWs to receive emotional support and provide feedback. Finally, seeking to address concerns related to confidentiality, we are enthusiastic that we were able to advertise this program as completely anonymous, since counselors are never made aware of user's personal information. Approximately 75% of program users were clinical HCWs and the assurance of anonymity and confidentiality may have contributed to this trend, since clinical HCWs are often very concerned about the confidentiality of mental health services and potential impacts of seeking such services on licensure (12, 13). A key lesson learned from the implementation of this program is the need for repeated, tailored outreach and messaging, since we experienced noticeable upticks in usage immediately following health system, department, or division-wide email and verbal virtual announcements. In addition to providing recurring reminders to our HCWs regarding emotional support, announcements were made on a staggered, rolling basis to ensure our counselors' capacity to provide sufficient support.

Based on the feedback we received from the online interactive screening program, we developed additional individual-level and institutional-level services, including an emotional support request phone line, embedded designated mental health clinicians, leadership development courses, and parenting forums. We also provided feedback in the larger institutional effort to launch community pods. At this time, the most utilized additional service has been the emotional support request line and among staff member callers, the proportion of HCWs with clinical or non-clinical duties has been fairly similar (40% non-clinical, 37% clinical, and 23% not specified). In addition, among women HCW callers, concerns have closely mirrored those identified in the interactive screening program. One of the most useful aspects of both the interactive screening program and the emotional support request line has been that, in addition to providing emotional support, counselors have been able to direct women HCWs to specific resources based on the concerns they raised. As is the case with large health systems, HCWs may seek support, but due to the fragmented nature of service development and hosting, many remain unaware of existing services that are available for use. By creating a centralized catalog for services and resources, we believe we were able to successfully direct HCWs to certain types of support they were seeking, but did not know existed. We began offering the leadership development courses for personnel managing and supervising non-clinical HCWs because many did not know how to best support their staff during crises, unlike leaders of clinical HCWs who have more experience supporting staff through stressful, adverse patient care outcomes. Although we piloted this service with non-clinical HCW leadership, based on positive testimonials, we hope to expand this offering institution-wide in the coming months. Finally, we anticipate high attendance for our upcoming parenting forums, since the themes of family/friends, work-life balance, and education, along with childcare, have consistently been cited by women HCWs.

Our work was made possible by utilizing a team-based approach and engaging HCWs and academic leaders with expertise in a variety of related disciplines, including disaster psychology, disaster behavioral health, peer support, and evaluation and delivery of mental health services to HCWs. Operating with workgroup members who have extensive experience in these fields enabled us to broaden the scope of our efforts and quickly mobilize to develop and provide additional support services, as requests from different HCW populations were made.

Compared to other mental health interventions for HCWs developed during the COVID-19 pandemic, as well as the Ebola and Severe Acute Respiratory Syndrome (SARS) outbreaks (15), our services were primarily focused on providing emotional support. Based on the review by Soklaridis et al. (15), while our intervention differed from others that increased availability to music therapy and group therapy sessions, our emotional support services did utilize aspects of other interventions that incorporated PFA and a warmline.

Several limitations of this perspective should be noted. Since our primary objective was to develop and introduce emotional support services to HCWs as quickly as possible, we were unable to measure women HCW well-being pre- and post-introduction of services. Additionally, the ratio of respondents to eligible clinical and non-clinical HCWs was not routinely tracked, as announcements of services were distributed on a regular basis to different groups within the health system. Finally satisfaction with services was not measured; however, as the testimonial at the beginning of this perspective indicates, we have received positive anecdotal feedback regarding our emotional support services.

## Recommendations

Based on our experience developing emotional support services for women HCWs during the COVID-19 pandemic, we recommend that institutions:

- Incorporate evidence-based disaster behavioral health models in emotional support and mental health initiatives for women HCWs.
- Leverage existing resources and the expertise of key institutional wellness stakeholders when developing support services.
- Develop a variety of services that address commonly cited barriers and allow women HCWs to engage with services that correspond to their level of comfort.
- Introduce multi-purpose interventions that provide immediate emotional support, as well as assess the needs of women HCWs to inform the development of additional services.
- Partner with institutional leadership to ensure a consistent flow of information pertaining to available support services, since utilization was dependent on continual announcements being disseminated.

As the COVID-19 pandemic persists and women HCWs continue to face occupational hazards, the demand for emotional support and mental health services is expected to remain high for quite some time. In fact, research from previous infectious disease outbreaks has found that the psychological footprint of crises, like the COVID-19 pandemic, disproportionately impacts women HCWs and has the potential to affect HCW mental health for years. As a result, institutions should be taking a longitudinal approach to planning and launching initiatives to support the mental health and well-being of women HCWs. We believe the process we used to develop and introduce emotional support services to women HCWs can be a helpful guide for organizations seeking to support their staff during the COVID-19 pandemic and beyond. Women HCWs are committed to managing their current and future professional, patient care, familial, and personal responsibilities. The COVID-19 pandemic has afforded us an opportunity to both rethink the way we support women HCWs and demonstrate institutional commitments to ensuring their mental health and well-being.

## Data Availability Statement

The original contributions presented in the study are included in the article/supplementary material, further inquiries can be directed to the corresponding author.

## Author Contributions

JS and KM wrote the first draft. AA conceptualized the graphic representation included in the manuscript. All authors contributed important editorial feedback, as well as read and approved the final manuscript.

## Conflict of Interest

The authors declare that the research was conducted in the absence of any commercial or financial relationships that could be construed as a potential conflict of interest.

## References

[1] RobinsonGE. Stresses on women physicians: consequences and coping techniques. Depress Anxiety. (2003) 17:180–9. 10.1002/da.1006912768652

[2] MullenK. Barriers to work–life balance for hospital nurses. Workplace Health Saf . (2015) 63:96–9. 10.1177/216507991456535525994973

[3] GuilleCFrankEZhaoZKalmbachDANietertPJMataDA. Work-family conflict and the sex difference in depression among training physicians. JAMA Intern Med. (2017) 177:1766–72. 10.1001/jamainternmed.2017.513829084311PMC5820732

[4] TempletonKBernsteinCASukheraJNoraLMNewmanCBurstinH. Gender-Based Differences in Burnout: Issues Faced by Women Physicians. (2019). Available online at: https://nam.edu/gender-based-differences-in-burnout-issues-faced-by-women-physicians/ (accessed August 26, 2020).

[5] TrockelMTHamidiMSMenonNKRoweSGDudleyJCStewartMT. Self-valuation: attending to the most important instrument in the practice of medicine. Mayo Clin Proc. (2019) 94:2022–31. 10.1016/j.mayocp.2019.04.04031543254

[6] McMurrayJELinzerMKonradTRDouglasJShugermanRNelsonK. The work lives of women physicians. J Gen Intern Med. (2000) 15:372–80. 10.1111/j.1525-1497.2000.im9908009.x10886471PMC1495474

[7] EssaryACBernardKSCoplanBDehnRForisterJGSmithNE. Burnout and Job and Career Satisfaction in the Physician Assistant Profession: A Review of the Literature. (2018). Available online at: https://nam.edu/burnout-and-job-and-career-satisfaction-in-the-physician-assistant-profession-a-review-of-the-literature/ (accessed August 26, 2020).

[8] BrandfordAAReedDB. Depression in registered nurses: a state of the science. Workplace Health Saf . (2016) 64:488–511. 10.1177/216507991665341530209987

[9] GrossCPMeadLAFordDEKlagMJ. Physician, heal thyself?: regular source of care and use of preventive health services among physicians. Arch Intern Med. (2000) 160:3209–14. 10.1001/archinte.160.21.320911088080

[10] Malachi JY. Physician assistants' preventive medicine practices and related habits, attitudes, and beliefs (dissertation). Walden University, Minneapolis, MN, United States (2015).

[11] DavisMDetreTFordDEHansbroughWHendinHLaszloJ. Confronting depression and suicide in physicians: a consensus statement. JAMA. (2003) 289:3161–6. 10.1001/jama.289.23.316112813122

[12] GoldKJAndrewLBGoldmanEBSchwenkTL. I would never want to have a mental health diagnosis on my record: a survey of female physicians on mental health diagnosis, treatment, and reporting. Gen Hosp Psychiatry. (2016) 43:51–7. 10.1016/j.genhosppsych.2016.09.00427796258

[13] CaresAPaceEDeniousJCraneLA. Substance use and mental illness among nurses: Workplace warning signs and barriers to seeking assistance. Subst Abus. (2015) 36:59–66. 10.1080/08897077.2014.93372525010597

[14] de PabloGSSerranoJVCatalanAArangoCMorenoCFerreF. Impact of coronavirus syndromes on physical and mental health of health care workers: Systematic review and meta-analysis. J Affect Disord. (2020) 275:48–57. 10.1016/j.jad.2020.06.02232658823PMC7314697

[15] SoklaridisSLinELalaniYRodakTSockalingamS. Mental health interventions and supports during COVID-19 and other medical pandemics: a rapid systematic review of the evidence. Gen Hosp Psychiatry. (2020) 66:133–46. 10.1016/j.genhosppsych.2020.08.00732858431PMC7442905

[16] LaiJMaSWangYCaiZHuJWeiN. Factors associated with mental health outcomes among health care workers exposed to coronavirus disease 2019. JAMA Netw Open. (2020) 3:e203976. 10.1001/jamanetworkopen.2020.397632202646PMC7090843

[17] PappaSNtellaVGiannakasTGiannakoulisVGPapoutsiEKatsaounouP. Prevalence of depression, anxiety, and insomnia among healthcare workers during the COVID-19 pandemic: a systematic review and meta-analysis. Brain Behav Immun. (2020) 88:901–7. 10.1016/j.bbi.2020.05.02632437915PMC7206431

[18] KangLMaSChenMYangJWangYLiR. Impact on mental health and perceptions of psychological care among medical and nursing staff in Wuhan during the 2019 novel coronavirus disease outbreak: a cross-sectional study. Brain Behav Immun. (2020) 87:11–7. 10.1016/j.bbi.2020.03.02832240764PMC7118532

[19] LiXYuHBianGHuZLiuXZhouQ. Prevalence, risk factors, and clinical correlates of insomnia in volunteer and at home medical staff during the COVID-19. Brain Behav Immun. (2020) 87:140–1. 10.1016/j.bbi.2020.05.00832380272PMC7198418

[20] LiGMiaoJWangHXuSSunWFanY. Psychological impact on women health workers involved in COVID-19 outbreak in Wuhan: a cross-sectional study. J Neurol Neurosurg Psychiatry. (2020) 91:895–7. 10.1136/jnnp-2020-32313432366684

[21] ÖzdinSBayrakÖzdin S. Levels and predictors of anxiety, depression and health anxiety during COVID-19 pandemic in Turkish society: the importance of gender. Int J Soc Psychiatry. (2020) 66:504–11. 10.1177/002076402092705132380879PMC7405629

[22] WangYDiYYeJWeiW. Study on the public psychological states and its related factors during the outbreak of coronavirus disease 2019 (COVID-19) in some regions of China. Psychol Health Med. (2020) 26:13–22. 10.1080/13548506.2020.174681732223317

[23] RossiRSocciVPacittiFDi LorenzoGDi MarcoASiracusanoA. Mental health outcomes among frontline and second-line health care workers during the coronavirus disease 2019 (COVID-19) pandemic in Italy. JAMA Netw Open. (2020) 3:e2010185. 10.1001/jamanetworkopen.2020.1018532463467PMC7256664

[24] MullerRAEStenslandRSØvan de VeldeRS. The mental health impact of the covid-19 pandemic on healthcare workers, and interventions to help them: a rapid systematic review. Psychiatry Res. (2020) 293:113441. 10.1016/j.psychres.2020.11344132898840PMC7462563

[25] López-AtanesMRecio-BarberoMSáenz-HerreroM. Are women still the other? Gendered mental health interventions for health care workers in Spain during COVID-19. Psychol Trauma. (2020) 12:S243–4. 10.1037/tra000075132538661

[26] MiottoKSanfordJBrymerMJBurschBPynoosRS. Implementing an emotional support and mental health response plan for healthcare workers during the COVID-19 pandemic. Psychol Trauma. (2020) 12:S165–7. 10.1037/tra000091832525378

[27] Committee on Post-Disaster Recovery of a Community's Public Health Medical and Social Services. Healthy, Resilient, and Sustainable Communities After Disaster: Strategies, Opportunities, and Planning for Recovery. Washington, DC: National Academies Press (2015). p. 476.26401544

[28] National Child Traumatic Stress Network. Psychological First Aid (PFA) Field Operations Guide: 2nd Edition. (2006). Available online at: https://www.nctsn.org/resources/psychological-first-aid-pfa-field-operations-guide-2nd-edition (accessed August 08, 2020).

[29] ShanafeltTRippJTrockelM. Understanding and addressing sources of anxiety among health care professionals during the COVID-19 pandemic. JAMA. (2020) 323:2133–4. 10.1001/jama.2020.589332259193

[30] KaufmanJStoddardJ. The Coronavirus Impact Scale. (2020). Available online at: https://disasterinfo.nlm.nih.gov/search/?source=2587 (accessed August 05, 2020).

[31] KroenkeKSpitzerRLWilliamsJBLöweB. An ultra-brief screening scale for anxiety and depression: the PHQ−4. Psychosomatics. (2009) 50:613–21. 10.1016/S0033-3182(09)70864-319996233

[32] KiselySWarrenNMcMahonLDalaisCHenryISiskindD. Occurrence, prevention, and management of the psychological effects of emerging virus outbreaks on healthcare workers: rapid review and meta-analysis. BMJ. (2020) 369:m1642. 10.1136/bmj.m164232371466PMC7199468

[33] VanGeestJBJohnsonTPWelchVL. Methodologies for improving response rates in surveys of physicians: a systematic review. Eval Health Prof . (2007) 30:303–21. 10.1177/016327870730789917986667

